The article "The Two-Component System CpxRA Negatively Regulates the Locus of Enterocyte Effacement of Enterohemorrhagic Escherichia coli Involving σ32 and Lon protease" was retracted in 2025. Reasons: duplicated images; concerns about the images.

# The Two-Component System CpxRA Negatively Regulates the Locus of Enterocyte Effacement of Enterohemorrhagic *Escherichia coli* Involving σ^32^ and Lon protease

**DOI:** 10.3389/fcimb.2016.00011

**Published:** 2016-02-05

**Authors:** Miguel A. De la Cruz, Jason K. Morgan, Miguel A. Ares, Jorge A. Yáñez-Santos, James T. Riordan, Jorge A. Girón

**Affiliations:** ^1^Unidad de Investigación Médica en Enfermedades Infecciosas y Parasitarias, Centro Médico Nacional Siglo XXI-IMSSMexico City, Mexico; ^2^Emerging Pathogens Institute, University of FloridaGainesville, FL, USA; ^3^Department of Cell Biology, Microbiology, and Molecular Biology, University of South FloridaTampa, FL, USA; ^4^Facultad de Estomatología, Benemerita Universidad Autonoma de PueblaPuebla, Mexico; ^5^Centro de Deteccion Biomolecular, Benemerita Universidad Autonoma de PueblaPuebla, Mexico

**Keywords:** CpxRA, Lon protease, sigma factor 32, LEE, EHEC

## Abstract

Enterohemorrhagic *Escherichia coli* (EHEC) is a significant cause of serious human gastrointestinal disease worldwide. EHEC strains contain a pathogenicity island called the locus of enterocyte effacement (LEE), which encodes virulence factors responsible for damaging the gut mucosa. The Cpx envelope stress response of *E. coli* is controlled by a two-component system (TCS) consisting of a sensor histidine kinase (CpxA) and a cytoplasmic response regulator (CpxR). In this study, we investigated the role of CpxRA in the expression of LEE-encoded virulence factors of EHEC. We found that a mutation in *cpxA* significantly affected adherence of EHEC to human epithelial cells. Analysis of this mutant revealed the presence of high levels of CpxR which repressed transcription of *grlA* and *ler*, the main positive virulence regulators of the LEE, and influenced negatively the production of the type 3 secretion system–associated EspABD translocator proteins. It is known that CpxR activates *rpoH* (Sigma factor 32), which in turns activates transcription of the *lon* protease gene. We found that transcription levels of *ler* and *grlA* were significantly increased in the *lon* and *cpxA lon* mutants suggesting that *lon* is involved in down-regulating LEE genes. In addition, the *Galleria mellonella* model of infection was used to analyze the effect of the loss of the *cpx* and *lon* genes in EHEC's ability to kill the larvae. We found that the *cpxA* mutant was significantly deficient at killing the larvae however, the *cpxA lon* mutant which overexpresses LEE genes *in vitro*, was unable to kill the larvae, suggesting that virulence in the *G. mellonella* model is T3SS independent and that CpxA modulates virulence through a yet unknown EHEC-specific factor. Our data provides new insights and broadens our scope into the complex regulatory network of the LEE in which the CpxA sensor kinase plays an important role in a cascade involving both global and virulence regulators.

## Introduction

Human infections with enterohemorragic *Escherichia coli* (EHEC) O157:H7 can cause diarrhea ranging from mild to bloody and can induce hemorrhagic colitis (Riley et al., 1983; Blattner et al., 1997; Jonson et al., 2005). Some patients with hemorrhagic colitis develop a severe complication known as the hemolytic uremic syndrome (HUS) that can lead to kidney failure, thrombocytopenia, and microangiopathic hemolytic anemia (Riley et al., 1983; Perna et al., 1998). Adult cattle, other farm animals, and wild animals are common reservoirs of many EHEC serotypes (Ferens and Hovde, 2011; Nguyen and Sperandio, 2012). Human infection occurs through acquisition of the bacteria via consumption of contaminated food (ground meat or vegetables), water, unpasteurized fruit juices, and milk (Cody et al., 1999; Crump et al., 2002).

Hallmarks of EHEC pathogenicity are their ability to produce one or two Shiga toxins (Stx1 and Stx2), which are responsible for the HUS (Karmali et al., 1983; Paton and Paton, 1998) and colonization of the gut mucosa leading to the development of intestinal attaching and effacing (AE) lesions (Nataro and Kaper, 1998). Most of the gene products required for the formation of AE lesions by EHEC are present in a pathogenicity island called the locus of enterocyte effacement (LEE). The LEE contains 41 genes and is organized into five main polycistronic operons designated LEE1-5 (Elliott et al., 1998), which code for components of a type 3 secretion system (T3SS) and numerous effector proteins (Nguyen and Sperandio, 2012). The regulation of the LEE of EHEC involves a complex regulatory network comprising virulence (Ler, GrlA, and GrlR) and global regulators such as Pch, H-NS, IHF, Hha, Fis, BipA, QseA, GrvA, EtrA, YhiEF, SdiA, among others (Mellies et al., 2007).

The Cpx envelope stress response of *E. coli* is controlled by a two-component system (TCS) consisting of a sensor histidine kinase (CpxA) that phosphorylates the CpxR cytoplasmic response regulator. CpxA senses a variety of stimuli (e.g., pH changes, overexpression of envelope proteins such as NlpE or P pilus subunits, and alterations in membrane) within the bacterial cell envelope (Danese et al., 1995; Nakayama and Watanabe, 1995; Snyder et al., 1995; Jones et al., 1997; Danese and Silhavy, 1998; Hung et al., 2001). Phosphorylated CpxR (CpxR-P) upregulates the expression of a considerable number of genes with devoted functions in the periplasm such as periplasmic protein folding and degradation factors (Danese et al., 1995; Danese and Silhavy, 1997) or beyond the periplasm (De Wulf et al., 2002; Price and Raivio, 2009). The Cpx proteins have been implicated in virulence of some Gram-negative bacterial pathogens. For example, CpxR regulates mutualism and pathogenesis of *Xenorhabdus nematophila* (Herbert et al., 2007) and CpxR positively regulates the main virulence factors of *Legionella pneumophila* (Gal-Mor and Segal, 2003; Altman and Segal, 2008). The absence of the sensor kinase affects the expression of virulence factors in many pathogens. CpxA was reported to be involved in pH-dependent regulation of VirF and HilA, central regulators of the invasion genes of *Shigella flexneri* and *Salmonella enterica* serovar Typhimurium, respectively (Nakayama and Watanabe, 1998; Nakayama et al., 2003). A Tn*phoA* insertion in the *cpxA* gene of *S*. Typhi reduced adherence and invasion to epithelial cells (Leclerc et al., 1998). Similarly, these phenotypes were significantly reduced in a *cpxA* mutant of *S*. Typhimurium that constitutively activated the Cpx pathway (Humphreys et al., 2004). Further, a *cpxA* mutant of *Yersinia pseudotuberculosis* was affected in type-3 secretion (Carlsson et al., 2007a,b) and the deletion of *cpxA* of *Hemophilus ducreyi* impaired its ability to infect humans (Spinola et al., 2010).

The CpxRA TCS has been also implicated in the regulation of enteropathogenic *E. coli* (EPEC) virulence factors (Vogt et al., 2010). The Cpx envelope stress response both facilitated and inhibited production of the EPEC bundle-forming pilus. In addition, an EPEC *cpxA24* mutant (affected in the phosphatase activity) inhibited T3S of translocators and effectors proteins by an unknown mechanism (Macritchie et al., 2008).

The function of the CpxRA TCS in the expression of LEE-associated virulence genes of EHEC has not been studied before. In this work, we investigated the role of the CpxRA TCS in intimate cell adherence and production of T3SS-associated determinants such as proteins associated with the EspA filament. We propose a model of how this TCS interplays with other known and unknown regulatory networks to modulate expression of virulence factors encoded in the LEE pathogenicity island.

## Materials and methods

### Bacterial strains and growth conditions

Bacterial strains and plasmids used in this study are listed in Table 1. Strains were routinely cultured with shaking at 37°C in Luria-Bertani (LB) broth (Difco) or Dulbecco's modified essential medium (DMEM) (Invitrogen). Ampicillin (50 μg/ml), kanamycin (50 μg/ml), and chloramphenicol (50 μg/ml) were added when required. To measure gene transcription and production of proteins overnight LB cultures were centrifuged and resuspended in fresh DMEM to an OD_600_ of 1. Then, 250 ml-flasks containing 50 ml of LB or DMEM were inoculated with 1 ml of the bacterial suspensions and incubated for 6 h at 37°C in a shaking incubator at 200 rpm. For induction of NlpE from plasmid pCA-NlpE, 50 μM IPTG was added to the growth medium 2 h post-inoculation. When plasmid pBAD-CpxA was used we did not induce *cpxA* expression from the arabinose promoter since the leaky expression that occurs is enough to complement the absence of CpxA in the chromosome.

**Table 1:** **Strains and plasmids used in this study**.

**Strains or plasmids**	**Genotype and/or relevant markers**	**References**
**K-12**		
MC4100	F' *araD139* Δ (*argF*-*lac*)*U169 rpsL150 relA1 flb5301 deoC1 ptsF25 rbsR*	Casadaban, 1976
**EHEC**		
EDL933 (O157:H7)	Wild-type strain	Riley et al., 1983
EDL933 Δ*cpxR*	Δ*cpxR*::Km^r^	This work
EDL933 Δ*cpxA*	Δ*cpxA*::Km^r^	This work
EDL933 Δ*cpxRA*	Δ*cpxRA*::Km^r^	This work
EDL933 Δ*lon*	Δ*lon*::Km^r^	This work
EDL933 Δ*cpxA* Δ*lon*	Δ*cpxA*::Km^r^ Δ*lon*::Cm^r^	This work
EDL933 Δ*ackA-pta*	Δ*ackA-pta*::Km^r^	This work
EDL933 Δ*cpxA* Δ*ackA-pta*	Δ*cpxA*::Km^r^ Δ*ackA-pta*::Cm^r^	This work
**PLASMIDS**		
pBAD-*myc*-HisA	Expression vector containing a C-terminal *myc* epitope tag and polyhistidine region; Ap^r^	Invitrogen
pBAD-CpxA	pBAD-*myc*-HisA-derived plasmid, carrying the EHEC *cpxA* gene under an arabinose promoter	This work
pCA24N	High-copy-number cloning vector; Cm^r^	Kitagawa et al., 2005
pCA-NlpE	*nlpE* cloned downstream of the IPTG inducible promoter on pCA24N	Kitagawa et al., 2005
pFPV25	GFP reporter fusion vector; Ap^r^	Valdivia and Falkow, 1996
*cpxR-gfp*	pFPV25 derivative containing the *cpxR* promoter region (500 bp upstream from translation start site)	This work
*rpoH-gfp*	pFPV25 derivative containing the *rpoH* promoter region (1000 bp upstream from translation start site)	This work
*ler-gfp*	pFPV25 derivative containing the *ler* promoter region (1000 bp upstream from translation start site)	This work
*grlRA-gfp*	pFPV25 derivative containing the *grlRA* promoter region (1000 bp upstream from translation start site)	This work
*nleA-gfp*	pFPV25 derivative containing the *nleA* promoter region (500 bp upstream from translation start site)	This work
pKD46	Lambda Red recombinase system under the arabinose promoter; Ap^r^	Datsenko and Wanner, 2000
pKD3	Plasmid containing the Cm cassette for Lambda Red Recombination; Ap^r^	Datsenko and Wanner, 2000
pKD4	Plasmid containing the Km cassette for Lambda Red Recombination; Ap^r^	Datsenko and Wanner, 2000

*Ap^r^, ampicillin resistance; Km^r^, kanamycin resistance; Cm^r^, chloramphenicol resistance*.

### Construction of isogenic mutants

Non-polar gene-deletion mutants were generated in the EHEC O157:H7 EDL933 wild-type strain by the lambda Red recombinase system (Datsenko and Wanner, 2000), using gene-specific primer pairs to amplify pKD4 kanamycin or pKD3 chloramphenicol-resistance genes as shown in Table 2.

**Table 2:** **Oligonucleotides used in this study**.

**Oligonucleotide**	**Sequence**	**Target gene**
**FOR GENE DELETION**		
cpxR-H1P1	TGC CTC GGA GGT ATT TAA ACA ATG AAT AAA ATC CTG TTA GTT GAT TGT AGG CTG GAG CTG CTT CG	*cpxR*
cpxR-H2P2	TGC GCG CGG TTA AGC TGC CTA TCA TGA AGC AGA AAC CAT CAG GTA CAT ATG AAT ATC CTC CTT AG	*cpxR*
cpxA-H1P1	CTA CCT GAT GGT TTC TGC TTC ATG ATA GGC AGC TTA ACC GCG CGC TGT AGG CTG GAG CTG CTT CG	*cpxA*
cpxA-H2P2	TCC TGC CTA CAA ATG CGG AGT TTA ACT CCG CTT ATA CAG CGG CAA CAT ATG AAT ATC CTC CTT AG	*cpxA*
lon-H1P1	TAG ATG GCG TGA AGC ACA GTC GTG TCA TCT GAT TAC CTG GCG GAA TGT AGG CTG GAG CTG CTT CG	*lon*
lon-H2P2	AGT GCA TTT TGC GCG AGG TCA CTA TTT TGC AGT CAC AAC CTG CAT CAT ATG AAT ATC CTC CTT AG	*lon*
ackA-H1P1	GTA TCA ATT ATA GGT ACT TCC ATG TCG AGT AAG TTA GTA CTG GTT TGT AGG CTG GAG CTG CTT CG	*ackA*
pta-H2P2	AAG CTG CGG ATG ATG ACG AGG TTA CTG CTG CTG CTG AGA CTG ATT CAT ATG AAT ATC CTC CTT AG	*pta*
**FOR TRANSCRIPTIONAL FUSIONS**		
cpxR-EcoRI-5′	GCG*GAATTC*TGCCATCTCAACCTG	*cpxR*
cpxR-BamHI-3′	TCA*GGATCC*AACAGGATTTTATTC	*cpxR*
rpoH-EcoRI-5′	GCG*GAATTC*TATTATCCGTCACCG	*rpoH*
rpoH-BamHI-3′	GCT*GGATCC*TGCATTTTGTCAGTC	*rpoH*
ler-EcoRI-5′	GAG*GAATTC*GCTTTCAGGAAAC	*ler*
ler-BamHI-3′	CAT*GGATCC*AATAAATAATCTCCGC	*ler*
grlRA-EcoRI-5′	ACC*GAATTC*TTAAAGGGGAGCGCCG	*grlRA*
grlRA-BamHI-3′	CTA*GGATCC*CCATCCTTCATAATC	*grlRA*
nleA-EcoRI-5′	CGC*GAATTC*ACACTACATTTAGAGTC	*nleA*
nleA-BamHI-3′	GAT*GGATCC*GTCGGTTGAATGTTC	*nleA*
**FOR GENE CLONING**		
cpxA-NcoI-5′	GCT*CCATGG*TAGGCAGCTTAACCGCG	*cpxA*
cpxA-HindIII-3′	CGG*AAGCTT*ACTCCGCTTATACAGC	*cpxA*

*Italic letters indicate the respective restriction enzyme site in the primer*.

### Construction of plasmids and *gfp* transcriptional fusions

*gfp* transcriptional fusions were generated by cloning PCR products corresponding to promoter regions into pFPV25 (see primers in Table 2). The PCR products were digested with *Eco*RI and *Bam*HI and ligated to pFPV25 previously digested with the same enzymes. For cloning of *cpxA*, specific primers containing the *Nco*I (5′)/*Hind*III (3′) restriction sites were used to obtain PCR products, which were digested with *Nco*I and *Hind*III and then ligated into pBAD-*myc*-HisA previously digested with the same restriction enzymes, generating pBAD-CpxA.

### Bacterial infection and adherence assays

Cultured HeLa epithelial cells were used in adherence assays as previously described (Girón et al., 2002). These cells were cultivated at 37°C under 5% CO_2_ atmosphere in polystyrene 24-well plates (CellStar) containing glass coverslips. For the adherence assay, cell monolayers at 60–80% confluency were washed and reconstituted with DMEM (Invitrogen). As inoculum, we used 10^8^ bacteria grown overnight in DMEM at 37°C. The cells were infected for 3 h, washed with PBS to remove unbound bacteria, and fixed with 2% formalin/PBS for 20 min. For quantitative assessment of bacterial adherence to epithelial cells (wild type vs. mutants), infected cell monolayers were treated with 1 ml of 0.1% Triton X-100 for 15 min. Following lysis, bacteria were quantified by plating out 10-fold dilutions of the bacterial suspensions. Quantifications were performed in triplicate on thRee different days, and the mean results were expressed as adhering CFUs. Statistical analysis was performed by using Student's *t* test.

### Immunofluorescence

Primary rabbit anti-EspA antibody was added 1:3000 in 10% horse serum to formalin-fixed cells for 1 h followed by the appropriate secondary Alexa-Fluor 488 conjugate (1:5000) for 1 h, washed, mounted on glass slides, and then visualized using an Axio Imager 1.0 Zeiss microscope as previously described (Girón et al., 2002).

### Western blotting

Whole-cell extracts of EHEC strains grown in DMEM at 37°C for 6 h were subjected to SDS-PAGE in 12% polyacrylamide gels and electroblotted onto nitrocellulose membranes (Millipore) as previously described (Garnett et al., 2012). After blocking with non-fat milk, the membranes were incubated with primary rabbit antibodies against EspA (1:5000), EspB (1:2000), EspD (1:2000) or mouse anti-DnaK (1:20,000). Goat anti-rabbit or anti-mouse IgG (Biomeda) conjugated to horseradish peroxidase (1:10,000) was used as secondary antibodies, and the reactions were visualized with chemiluminescence reagents (Perkin Elmer).

### Quantitative real-time PCR (qRT-PCR)

RNA purification, cDNA synthesis, primers, qRT-PCR cycling conditions and data analysis followed previously described protocols (Riordan et al., 2010; Neupane et al., 2011). Bacterial cultures were grown to OD_600_ = 1.2 before RNA extraction (RNeasy™ kit, Qiagen, Valencia, CA) and cDNA synthesis (iScript, Bio-Rad, Carlsbad, CA). Quantitative real-time PCR (qRT-PCR) was performed using primers for *rrsH* (16S rRNA gene) to normalize cDNA levels. Reaction conditions included 40 cycles of denaturing at 94°C for 15-s, followed by annealing at 55°C for 20-s. Experiments were performed in triplicate on three different days and the results shown are the mean of the data produced.

### Flow cytometry analysis of bacteria grown in DMEM

Bacteria grown in DMEM were treated and analyzed by flow cytometry as previously described (De la Cruz et al., 2013). Bacteria were washed twice with PBS and immediately fixed in two volumes of 3% paraformaldehyde for 1 h. For flow cytometric analysis, bacteria were gated in FL2 and analyzed for the expression of GFP in FL1. Data were acquired with a FACSCalibur (BD Biosciences) and analyzed with the FlowJo software (Tree Star Inc., Ashland, OR). Experiments were performed in triplicate on three different days and the results shown are the mean of the data produced.

### Invertebrate virulence assays using *Galleria mellonella*

Virulence assays were performed as previously described (Leuko and Raivio, 2012; Morgan et al., 2014). Assays for virulence in *G. mellonella* were performed using 5th instar larvae purchased from GeorgiaCrickets.com. Upon arrival, all larvae were stored on wood chips in a 4°C refrigerator, and were used within 2 weeks of receipt. For survival assays, 10 larvae between 2- and 2.5-cm were selected for use for injection into each strain tested, and only larvae free of melanization (dark spots) or injury were used in experimentation. Bacterial cultures for virulence assays were grown to an OD_600_ = 0.5 in DMEM for induction of virulence genes. At the desired optical density, 1 mL of culture was pelleted by centrifugation in a 1.5 mL Eppendorf tube and washed twice with 10 mM MgSO_4_. For survival assays, 5 μL of a bacterial suspension containing 10^5^ CFUs were injected into the larval hemolymph through last left proleg using a 10 μl Hamilton syringe (26s gauge, 51 mm length, point style #2, cat. 80366). Following injection, larvae were placed in a sterile petri dish and incubated in the dark at 37°C for 96 h. Each assay contained a control group of larvae, which were either not injected, or injected with sterile 10 mM MgSO_4_. In each case, no control larvae were killed during the course of experimentation. No assays were performed beyond 96 h, as larvae began to form pupa beyond that time. At each assay time point, the number of larvae was scored as dead if they did not respond to touch. The % survival was calculated from 10 larvae as the 100% These experiments were performed were repeated three times on different days and the results shown are the mean of the data produced. When plasmid pBAD-CpxA was used we did not induce *cpxA* expression from the arabinose promoter since the leaky expression that occurs is enough to complement the absence of CpxA in the chromosome.

## Results

### Disruption of CpxRA affects adherence of EHEC to hela cells

We began this study by generating single and double mutants in the *cpxA* and *cpxR* genes in EHEC O157:H7 prototypic strain EDL933. To evaluate the role of these genes in bacterial adherence, we infected HeLa cell monolayers with the wild-type strain and derivative isogenic *cpx* mutants to quantify and compare adherence levels. Interestingly, the *cpxA* mutant was dramatically impaired in adherence (~100-fold) as compared to the wild-type strain or the *cpxA* mutant complemented with plasmid pBAD-CpxA (Figure 1A). In contrast, the single *cpxR* and the double *cpxRA* mutants were not affected in adherence to HeLa cells, indicating that the reduction of adherence noted in the *cpxA* mutant was CpxR-dependent (Figure 1A). These data were supported with light microscopy observations of HeLa cells infected with EHEC strains (Figure 1B). As shown, the *cpxA* mutant was poorly adherent to these cells in comparison to EDL933. We suspected that the mutation in *cpxA* could have impacted transcription of *cpxR*, thus we sought to determine transcription levels of *cpxR* using a *cpxR-gfp* fusion transformed in the wild-type strain and in *cpx* derivative mutants. In the absence of CpxR, the expression of the *cpxR-gfp* fusion diminished 5-fold (Figure 2A) as compared to expression in the wild-type strain. This result is in agreement with previous reports on the positive auto-regulation of *cpxR* (De Wulf et al., 1999; Price and Raivio, 2009). In contrast, high levels (3.2-fold) of *cpxR* transcription were seen in the *cpxA* mutant with respect to the wild-type strain (Figure 2A), suggesting that the reduced adherence of the *cpxA* mutant to human epithelial cells observed in Figure 1 was due to high production levels of CpxR, which most likely exerted negative regulation on a yet unknown factor. To support these transcriptional data, we then assessed the production of both CpxR and CpxA proteins in the *cpx* mutants by Western blotting (Figure 2B). In correlation with the transcriptional data we found that the CpxR response regulator was abundantly detected in the *cpxA* mutant (Figure 2B). As expected, CpxR was not detected in the *cpxR* mutant or the *cpxRA* double mutant. The mutation in *cpxR* also affected the production of the CpxA protein since no CpxA was found in these mutants (Figures 2A,B). It was previously reported that in the absence of the CpxA kinase sensor, CpxR can be phosphorylated with an acetyl phosphate produced by the acetate kinase (AckA) and phosphotransacetylase (Pta) enzymes (Batchelor et al., 2005; Spinola et al., 2010; Liu et al., 2012). To determine if the AckA-Pta pathway was responsible for the high level of *cpxR* transcription in the absence of CpxA, we measured the activity of the *cpxR-gfp* fusion in the wild-type strain and *ackA-pta* and *cpxA ackA-pta* mutants. Indeed, acetyl phosphate produced by the AckA-Pta pathway phosphorylated CpxR, rendering CpxR-P and activating the expression of *cpxR-gfp* fusion (Figure 2C).

**Figure 1:** **CpxA kinase sensor is required for EHEC adherence. (A)** Quantification of bacterial adherence to human cells. The indicated strains were incubated with HeLa cells for 3 h and the adherent bacteria expressed as CFUs after plating serial dilutions. The data are representative of a least three experiments performed in triplicate. **(B)** Giemsa staining of HeLa cell monolayers infected for 3 h with EHEC EDL933 (A), Δ*cpxR* (B), Δ*cpxA* (C), Δ*cpxA* (pBAD-CpxA) (D), Δ*cpxRA* (E). Adherence of the *cpxA* mutant is statistically significant with respect to that shown by the WT strain ^**^p < 0.01.

**Figure 2:** **High levels of CpxR expression in Δ***cpxA***. (A)** Expression of *cpxR* is derepressed in the absence of CpxA. EHEC wt (EDL933) and various *cpx* mutants carrying a transcriptional fusion *cpxR-gfp* were grown in DMEM and samples were taken at 6 h post-inoculation. The relative fluorescence intensity of bacteria was determined by flow cytometry. Between 5000 and 10,000 bacteria were analyzed to calculate the mean GFP/bacterium. **(B)** CpxR and CpxA proteins were analyzed by Western Blotting in wild-type and *cpx* derivative mutants. Samples were taken at 6-h post-inoculation and were used anti-CpxR and anti-CpxA antibodies. **(C)** High expression of *cpxR* in the absence of CpxA is dependent on both AckA and Pta enzymes. EHEC wt (EDL933) and various *ackA-pta* mutants carrying a transcriptional fusion *cpxR-gfp* were grown in DMEM and samples were taken at 6 h post-inoculation. **(D)** Quantification of bacterial adherence upon overexpression of NlpE. The indicated strains were incubated with HeLa cells for 6 h and the adherent bacteria expressed as CFUs after plating serial dilutions. NlpE was overexpressed with 50 μM IPTG. The data are representative of a least three experiments performed in triplicate. Adherence statistically different with respect to that shown by the WT strain (^*^p < 0.05; ^**^p < 0.01).

We were intrigued as to why high levels of CpxR were responsible for affecting the adherence of the *cpxA* mutant. It is known that when the NlpE lipoprotein is overexpressed in *E. coli* K-12 it triggers a Cpx response (Snyder et al., 1995). Thus, we overexpressed NlpE lipoprotein from an inducible plasmid transformed in the wild-type strain and the *cpxR* mutant (Figure 2D). It was found that the overexpression of NlpE in the wild-type strain led to a 100-fold reduction in adherence while no effect was seen in the *cpxR* mutant either with normal or high levels of NlpE (Figure 2D), indicating that overexpression of CpxR is responsible for the reduction in adherence levels.

### CpxRA regulates negatively the expression of EspABD translocator proteins

Intimate cell adherence of EHEC is dependent on the expression of intimin and T3SS-associated proteins Tir (translocated intimin receptor), EspA (T3S filament protein), and EspB and EspD (filament tip-associated proteins) encoded in the LEE5 operon (Ebel et al., 1998; Kresse et al., 1999; Schüller and Phillips, 2010). A previous study showed that the expression of LEE5 of EPEC was reduced in a *cpxA24* background (Macritchie et al., 2008). This *cpxA24* mutant was affected in the phosphatase activity but not in its auto-phosphorylation and kinase activities, resulting in high concentration levels of CpxR-P (Raivio and Silhavy, 1997). Given that we showed above that a *cpxA* mutant of EHEC was significantly affected in adherence to human cells (Figure 1), in this study, we sought to investigate the role of CpxA in the function of the T3SS of EHEC by testing the *cpxA* null mutant constructed here in gene expression and production of T3SS products. This *cpxA* null mutant exhibited high levels of *cpxR* transcripts (Figure 2A) and overproduced CpxR (Figure 2B). We analyzed production of EspA, EspB, and EspD proteins in the wild-type strain and the *cpx* mutants growing in DMEM. Of all the strains tested only the *cpxA* mutant showed a significant decrease in production of these translocator proteins (Figure 3A). These data explained with great level of certainty the initial observations of the diminished adherence of the *cpxA* mutant (Figure 1). The *cpxA* mutant complemented with the pBAD-CpxA plasmid restored production of EspA, EspB, and EspD. The *cpxRA* double mutant had a similar adherence phenotype as the wild-type strain (Figure 3A). We wanted to know if high levels of NlpE affected the production of the EspABD proteins via activation of the Cpx TCS. We found that activation of Cpx by overexpression of NlpE negatively affected the production of the EspA filament and EspB and EspD tip-associated proteins in the wild-type strain, but not in the absence of CpxR (e.g., in the *cpxR* mutant), suggesting that high levels of CpxR repressed the expression of translocator proteins genes (Figure 3B). Our data are in agreement with a report by Macritchie et al. (2008), which showed that overexpression of NlpE leads to repression of EspA, EspB, and EspD secretion (34). We sought to investigate if this repression occurred at transcriptional level, thus we measured *espA* transcription by quantitative Real-Time PCR (qPCR). As predicted, *espA* transcriptional expression was dramatically diminished (72.6-fold) in the absence of CpxA (Table 3). Immunofluorescence microscopy experiments employing anti-EspA antibodies ultimately confirmed that the EspA filament typically seen in the wild type strain (Figures 4A,B) was absent in the *cpxA* mutant during EHEC infection of HeLa cells (Figure 4C). The production of the EspA filament was restored in the complemented strain (Figure 4D). Our data support the notion that high levels of CpxR negatively controls EHEC adherence to human cells, diminishing both production and secretion of the translocator proteins, and in particular the formation of the EspA filament. All together, the data obtained with the *cpxA* and the *cpxRA* mutants indicate that a functional CpxRA TCS is required for proper function of the T3SS.

**Figure 3:** **Translocator proteins are reduced in a ***cpxA*** mutant**. EspA, EspB, and EspD proteins were analyzed by Western Blotting in wild-type and *cpx* derivative mutants **(A)** or under NlpE overexpression (50 mM IPTG) in the wt and *cpxR* mutant **(B)**. Samples were taken at 3-h post-inoculation and anti-EspA, anti-EspB, and anti-EspD antibodies were used for detection of Esps.

**Table 3:** **Transcript levels of LEE genes in the absence of CpxA**.

**Gene**	**wt/*cpxA***
*ler*	13.4 (1.32)
*grlA*	8.18 (0.56)
*espA*	72.63 (9.87)
*tir*	2.94 (0.12)

*Transcript levels were determined by qRT-PCR in triplicate in three different days. The data shown are the mean of the data produced. Repression levels of ler, grlA, espA, and tir in the cpxA mutant with respect to the wild-type strain. Transcript levels were normalized to the rrsH ribosomal gen (16S rRNA)*.

**Figure 4:** **T3SS is affected in the absence of CpxA**. Immunofluorescence of HeLa cells infected with **(A)** EHEC strain EDL933, **(B)** high magnification of panel A, **(C)** *cpxA* mutant, and **(D)** complemented *cpxA* mutant using anti-EspA antibody. EspA filaments are shown in green and bacteria and eukaryotic cells DNA was stained red with propidium iodine.

### High levels of CpxR repress the ler-regulon

To explore if CpxR regulates other genetic elements contained in the LEE of EHEC, we performed qPCR experiments to analyze the level of expression of several genes encoded in the different LEE operons and in particular of the positive virulence-associated regulators *ler* and *grlA*. To achieve this, we constructed *gfp* fusions harboring promoter regions of each of these genes. We targeted expression of two positive transcriptional regulators *ler* and *grlA* contained in the LEE and the translocated intimin-receptor *tir*. Interestingly the expression of *ler* (13.4-fold), *grlA* (8.18-fold) and *tir* (2.94-fold) were diminished in the absence of CpxA with respect to the wild-type strain (Table 3). In addition, we generated *gfp* transcriptional fusions with *ler, grlRA* and a non-LEE encoded effector A (*nleA)* genes. In agreement with the qPCR data the levels of *ler* (3.5-fold) and *grlA* (3-fold) genes were repressed in the Δ*cpxA* mutant when compared to the wild type-strain confirming that high levels of CpxR-P repressed the LEE (Figure 5A). The *nleA* gene, which is located outside the LEE but whose expression is Ler-dependent, was also repressed in the *cpxA* mutant (Figure 5B). The absence of CpxR did not affect the expression of *ler, grlRA*, and *nleA* genes since similar values of transcription were found between wild-type strain and the *cpxR* and *cpxRA* mutans (data not shown). These results indicate that high levels of CpxR seen in the absence of CpxA sensor kinase represses the Ler-regulon in EHEC as well as virulence genes outside the LEE.

**Figure 5:** **RpoH-Lon pathway represses LEE. (A)** Expression of *ler-gfp, grlRA-gfp*, and *nleA-gfp* are derepressed in the absence of Lon. EHEC wt (EDL933), Δ*cpxA*, Δ*lon*, and Δ*cpxA* Δ*lon* carrying transcriptional fusions *ler-gfp, grlRA-gfp*, and *nleA-gfp* were grown in DMEM and samples were taken at 6 h post-inoculation. **(B)** Expression of *rpoH-gfp* is derepressed in the absence of CpxA. EHEC wt (EDL933) and various *cpx* mutants carrying a transcriptional fusion *rpoH-gfp* were grown in DMEM and samples were taken at 6 h post-inoculation. The relative fluorescence intensity of bacteria was determined by flow citometry. Between 5000 and 10,000 bacteria were analyzed to calculate the mean GFP/bacterium. Transcript levels of *espA* were determined by qPCR in the wt, Δ*cpxA*, Δ*lon*, and Δ*cpxA* Δ*lon* **(C)** under NlpE overexpression (50 μM IPTG) in the wt and *lon* mutant **(D)**. Transcript levels were normalized to the *rrsH* ribosomal gen (16S rRNA). Expression statistically different with respect to that shown by the WT strain (^*^p < 0.05; ^**^p < 0.01; ^***^p < 0.001; ns, not significant).

### Lon is required for repression of the LEE in the absence of CpxA

To provide insights into the mechanism of LEE repression in the absence of CpxA, we monitored transcriptional levels of regulatory genes, which are known to be modulated by the CpxRA regulon. The *rpoH* gene, which codes for Sigma factor 32 (σ^32^), was reported to be activated by CpxR in *E. coli* K-12 (Zahrl et al., 2006). To demonstrate that CpxR activates the *rpoH* gene in EHEC, we measured *rpoH* transcription levels using a *rpoH*-*gfp* transcriptional fusion in the wild-type and *cpx* mutant backgrounds. In agreement with Zahrl et al. (2006), *rpoH* expression was diminished in the absence of CpxR (Figure 5B). Interestingly, *rpoH-gfp* transcription levels were increased 3-fold in the *cpxA* mutant (Figure 5B), indicating that high levels of CpxR in this mutant enhanced *rpoH* transcription. We were unable to delete *rpoH* in EHEC EDL933 strain by the λRed recombination method probability because of its deleterious effect (Datsenko and Wanner, 2000). In *E. coli* K-12, σ^32^ regulates genes involved in heat-shock response such as transcriptional regulators, chaperone-assisted protein folding catalysts, DNA modification, and transporters, amongst others (Nonaka et al., 2006). The *lon* gene codes for the Lon protease and is one of the genes most affected by σ^32^ (Zhao et al., 2005; Nonaka et al., 2006). Even when *rpoH* transcription was stimulated in the absence of CpxA, *lon* transcripts were not affected in a *cpxA* mutant (data not shown). To evaluate the role of Lon in LEE expression we quantitated transcription levels of *ler, grlA*, and *nleA* genes in a *lon* mutant by measuring activity of *gfp* fusions (Figure 5A). Surprisingly, in contrast to the wild-type strain and the *cpxA* mutant, the expression of these genes was derepressed in the *lon* and the *lon cpxA* mutants as they exhibited high levels of *gfp* activity (Figure 5A). These results strongly indicate that the repression of *ler, grlA*, and *nleA* genes in the *cpxA* mutant was Lon-dependent. To corroborate the role of Lon in the Cpx-mediated repression, we analyzed *espA* expression by qRT-PCR. Transcription of the *espA* gene was up-regulated in both the *lon* single mutant (4-fold) and the *cpxA lon* double mutant (7-fold) as compared to the wild-type strain (Figure 5C). Moreover, we overexpressed the NlpE lipoprotein in both the wild-type and the *lon* mutant backgrounds and found that *espA* was repressed 8.7-fold in the wild-type strain and 1.8-fold in the *lon* mutant (Figure 5D). Based on our experimental data, we would propose a model supporting the existence of a complex regulatory CpxA-CpxR-RpoH-Lon-LEE cascade, involving a TCS, sigma factors, and a protease that act in concert to regulate virulence in EHEC (Figure 6). In this model, environmental signals and even perhaps host signals induce the phosphorylation of the CpxR protein which in turn activates σ^32^ leading to the expression of the *lon* gene and whose product would degrade regulatory proteins Ler and GrlA halting expression of the LEE or affecting the stability of others proteins that activate the Ler/GrlA circuit such as Pch's, GrvA, QseA, Fis, IHF, or BipA, and thus finally controlling virulence of EHEC.

**Figure 6:** **CpxA-CpxR-RpoH-Lon-LEE complex regulatory cascade**. Current model about the LEE regulation initiated by the CpxRA. CpxA senses a variety of stimulus (pH changes, copper, overexpression of envelope proteins such as NlpE or P pilus subunits, and alterations in membrane) within the bacterial cell envelope (Danese et al., 1995; Nakayama and Watanabe, 1995; Snyder et al., 1995; Jones et al., 1997; Danese and Silhavy, 1998; Hung et al., 2001; Yamamoto and Ishihama, 2005). *rpoH* P1 promoter (Sigma 32 factor) is activated by CpxR (Figure 5A, Zahrl et al., 2006) and RpoH activates *lon* promoter (Zhao et al., 2005; Nonaka et al., 2006). Lon negatively regulates LEE expression probably affecting stability of Ler and/or GrlA proteins (Figure 5).

### CpxA is required for virulence of EHEC in the *Galleria mellonella* infection model

The ability of EHEC to cause intestinal pathology is attributed in part to the expression of LEE genes in the host gut environment (Garmendia et al., 2005; Melton-Celsa et al., 2012; Lewis et al., 2014). Given that the EHEC *cpxA* mutant showed diminished expression of LEE genes (Figure 5A, Table 3) we sought to investigate the role of the CpxRA TCS in EHEC's virulence in the *Galleria mellonella* larvae model. This model has been employed to measure virulence of *Salmonella*, EPEC, and other enteric and non-enteric pathogens (O'Loughlin et al., 2010; Debnath et al., 2013; Bontemps-Gallo et al., 2015; De la Cruz et al., 2015; Thomassin et al., 2015). We compared the ability of EHEC strains (wild-type vs. mutants) to kill *G. mellonella* larvae. We injected 10 larvae with 10^5^ CFU/ml of each strain tested and % survival was recorded after 24, 48, 72, and 96 h of infection. The experiments were repeated three times on three different days. We found that the mutation in *cpxA* resulted in a significant reduction in virulence since only 20% (2 out of 10) of the larvae survived as compared to the wild-type strain after 96 h of infection (Figure 7). The *cpxA* mutant complemented with the pBAD-CpxA plasmid restored virulence to levels similar to the wild-type strain. The single *cpxR* and double *cpxRA* mutants did not show attenuation in virulence and most importantly were more virulent than the wild-type strain (Figure 7). These data support a negative role of CpxR in the regulation of virulence of EHEC in this *in vivo* model of infection. Our transcriptional data showed that the Lon protease is involved in a transcriptional complex cascade that initiates with CpxA. To determine the role of Lon and CpxA in EHEC's virulence using the *G. mellonella* model, single and double mutants in the *cpx* and *lon* genes were evaluated. The *lon* single mutant had a slight attenuation in virulence with respect to the wild-type strain mainly at 24 and 48 h post-inoculation (Figure 7). Interestingly, the *cpxA lon* double mutant had a similar virulence behavior as the *cpxA* mutant throughout the infection time frame, in spite of the high levels of LEE transcription previously seen in this mutant (Figure 5A). The fact that the single *cpxA* and *lon* mutants as well as the double *cpxA lon* mutants showed attenuation of virulence to different extent in the *G. mellonella* model confirms that the CpxA sensor kinase plays a crucial role in regulating CpxR-P levels, which are important for modulation of Lon and for maintaining virulence of EHEC.

**Figure 7:** **A ***cpxA*** mutant in EHEC is attenuated in the virulence by using ***G. mellonella*** model**. Survival of *G. mellonella* infected with 10^5^ cells of EHEC wt, Δ*cpxA*, Δ*cpxA* pBAD-CpxA, Δ*cpxR* and Δ*cpxRA*, Δ*lon* and Δ*cpxA* Δ*lon* was monitored for up to 4 days. Results represent the means from three independent experiments. See text for experimental details.

## Discussion

A growing number of studies implicate the CpxRA TCS in the virulence of numerous Gram-negative bacteria (O'Loughlin et al., 2010; Debnath et al., 2013; Bontemps-Gallo et al., 2015; De la Cruz et al., 2015; Thomassin et al., 2015). The present study describes the importance of the CpxA sensor kinase in the regulation of virulence of EHEC by modulating LEE expression. The absence of CpxA led to diminished production of T3SS translocator proteins (EspA, EspB, EspD) (Figure 3A). NlpE is a lipoprotein that activates the Cpx signal transduction pathway when it is overproduced (Snyder et al., 1995). We found that when NlpE is overexpressed in EHEC, adherence to human cells (Figure 2D) was significantly reduced probably due to down-regulation of translocator proteins, which are necessary to form the filament that is required for initial adherence mediated by Tir and intimin (Figure 4). More importantly, this negative effect in transcription and production of T3SS was due to low levels of transcription of the main positive regulators of LEE, *ler*, and *grlA* (Table 3, Figure 5A) (Mellies et al., 1999; Bustamante et al., 2001; Deng et al., 2004; Barba et al., 2005).

In addition to their kinase activity, sensor kinases have phosphatase activity maintaining controlled levels of phosphorylation of their cognate response regulators (Kenney, 2010). In the absence of the CpxA phosphatase activity (e.g., in the *cpxA* mutant), phosphorylation of CpxR occurs by acetyl-phosphate produced by the AckA and Pta enzymes, causing high levels of CpxR-P (Batchelor et al., 2005; Wolfe et al., 2008; Liu et al., 2011; De la Cruz et al., 2015). In *E. coli* K-12, CpxR activates expression of Sigma factor 32 (*rpoH*) by controlling its P1 promoter (Zahrl et al., 2006). RpoH is associated with the heat-shock response and regulates numerous genes involved in metabolism and transport, among others. Moreover, RpoH has been reported to regulate virulence in several pathogens (Bang et al., 2005; Delory et al., 2006; Grall et al., 2009). One target of RpoH is the *lon* gene, which encodes a protease with pleiotropic functions in many pathogens (Wright et al., 1996; Robertson et al., 2000; Bretz et al., 2002; Takaya et al., 2005; Bertani et al., 2007). We found that high levels of CpxR-P activated the *rpoH* gene in EHEC but did not affect the *lon* transcription (Figure 5B, data not shown). Similar to what we found in our study, CpxR negatively regulated *Salmonella* SPI-1 by involving Lon protease, which specifically degraded HilD, a positive virulence regulator (Matsui et al., 2008; De la Cruz et al., 2015). By transcriptional fusions and qRT-PCR, we found that an EHEC *lon* mutant showed high levels of expression of *ler, grlA, espA*, and *nleA* genes (Figure 5A) suggesting that Lon down-regulates the activity of these virulence genes. Interestingly, the EHEC *lon cpxA* double mutant also showed high transcriptional levels of *ler, grlA, espA*, and *nleA* genes indicating that the repression seen in the *cpxA* single mutant was Lon-dependent (Figures 5B,C). The role of Lon in the Cpx-mediated repression was confirmed by overexpressing the NlpE lipoprotein and analyzing *espA* transcription in the wild-type and *lon* background. The overexpression of NlpE lipoprotein presented a slight negative effect in a *lon* mutant (Figure 5D). The same phenomenon was observed on the SPI-1 pathogenicity island in *S*. Typhimurium (De la Cruz et al., 2015), suggesting that Lon protease shows similar mechanisms of virulence repression in both pathogens. Thus, Lon regulates negatively the T3SS of EHEC, an activity also reported for *Salmonella enterica* and *Pseudomonas syringae* (Bretz et al., 2002; Takaya et al., 2005).

This cascade would be similar to the *cpxA24* phenotype described for EPEC (Macritchie et al., 2008). This inhibitory effect on LEE transcription was reported to be independent of EPEC-specific regulators because it was seen in both pathogenic and non-pathogenic strains of *E. coli*. Our data indicate that global regulators conserved in non-pathogenic *E. coli* such as Sigma factor 32 and Lon protease participate in regulation of the LEE. LEE repression via CpxRA involves a complex regulatory cascade comprising different regulatory proteins such as sigma factors, proteases and transcriptional regulators (Figure 6). The mechanism of Lon-mediated repression of LEE transcription is unknown. Recently, it was reported that Lon protease is necessary in the CpxR-mediated SPI-1 repression by affecting the stability of HilD, the central regulator of SPI-1 (De la Cruz et al., 2015). One possibility is that in EHEC, Lon affects the stability of Ler and GrlA positive regulators or alternatively that Lon degrades a positive regulator, which in turn activates the *ler*-*grlA* positive-feedback loop.

The importance of CpxA in the regulation of virulence factors has been described in detail for *Y. pseudotuberculosis* (Carlsson et al., 2007a,b; Liu et al., 2011, 2012). Similar to what we found here in EHEC, the null *cpxA* mutant was defective in the production of T3SS effector proteins (Carlsson et al., 2007a,b). CpxR-P directly represses transcription of *rovA*, the main positive regulator of the virulence of *Y. pseudotuberculosis* (Carlsson et al., 2007b). The mechanism of CpxR-mediated repression on EHEC T3SS is more complex and would involve both transcriptional and post-translational factors. CpxRA would sense specific signals present in the context of host infection (e.g., pH changes, misfolded proteins, metals, bacteria-cell contact) by activating Sigma factor 32 and Lon protease (Figure 6). Similar to *S*. Typhimurium (De la Cruz et al., 2015), Lon appears to be a crucial component in the virulence of several pathogens having as targets keys transcriptional regulators.

*G. mellonella* is an animal model used to study the virulence of many pathogens such as *P. aeruginosa* (Jander et al., 2000), *Campylobacter jejuni* (Senior et al., 2011), *Y. pseudotuberculosis* (Champion et al., 2009), *Acinetobacter baumannii* (Peleg et al., 2009), *Burkholderia cepacia* (Seed and Dennis, 2008), *L. monocytogenes* (Mukherjee et al., 2010), EPEC (Leuko and Raivio, 2012), *K. pneumoniae* (Insua et al., 2013), and *Salmonella* (Bender et al., 2013). In this study, we used the *G. mellonella* infection model to show that the mutation in *cpxA* significantly altered the ability of EHEC to infect this invertebrate rendering it attenuated in virulence. In our *in vitro* experiments, we were unable to find a phenotype for the *cpxR* and *cpxRA* mutant. However, using the *G. mellonella in vivo* model, we found that both the *cpxR* and *cpxRA* mutants were more virulent than the wild-type strain supporting the idea that CpxR is a negative regulator of EHEC virulence. In spite of the high levels of LEE transcription displayed by the *cpxA lon* double mutant (Figure 5A), this mutant remained avirulent in the *G. mellonella* model (Figure 7). It is possible that expression of other EHEC-specific virulence factors is affected in this mutant, such as the Shiga toxin, hemolysin, and EspP enterotoxin. Recently, it was been reported that an EHEC *cpxA* mutant was impaired in growth when cultured with glycerol-3-phosphate or glucose-6-phosphate as a sole carbon source and was outcompeted by the parent strain, even in nutrient-rich medium (Kurabayashi et al., 2014). Moreover, an EPEC-derived strain carrying a *cpxA24* gene, was attenuated in the virulence in *G. mellonella* due to its inability to survive and proliferate in hemolymph or to live in the whole larvae and to the diminished ability of the larvae to produce antimicrobial peptides such as cecropin and gloverin when infected with the bacteria (Leuko and Raivio, 2012). For comparison, only 35% of the larvae survived in the EHEC *cpxA* as compared to the wild-type strain after 72 h of infection, while in EPEC *cpxA24* 40% of the larvae survived at the same time of infection (Leuko and Raivio, 2012), indicating similarities between these two pathotypes in the *G. mellonella* model. However, the contribution of the T3SS in virulence using the *G. mellonella* model seems to be different between EPEC and EHEC: while in EPEC an *escN* mutant was attenuated (Leuko and Raivio, 2012), in EHEC the absence (*escN*) or overexpression (*grlR*) of T3SS did not significantly alter virulence (Morgan et al., 2014). Although our *in vivo* data supports a role for CpxA in the regulation of EHEC's virulence factors, it is important to note that the CpxRA TCS has pleiotropic regulatory effects on different bacterial genes. Our results show the transcriptional communication between global and specific regulators in EHEC. The effect of CpxRA on EHEC is an example of the complexity of a regulatory cascade that allows the spatiotemporal and coordinated expression of virulence factors during infection (Figure 6).

## Author contributions

Conceived and designed the experiments: MD and JG. Performed the experiments: MD, JM, and MA. Analyzed the data: MD, JM, JR, JY, and JG. Wrote the paper: MD and JAG.

### Conflict of interest statement

The authors declare that the research was conducted in the absence of any commercial or financial relationships that could be construed as a potential conflict of interest.
